This article has been retracted.

# Differentiation Between Humic and Non-Humic Substances Using Alkaline Extraction and Ultraviolet Spectroscopy

**DOI:** 10.1093/jaoacint/qsad001

**Published:** 2023-01-04

**Authors:** Lawrence Mayhew, Amit Pratap Singh, Peng Li, E Michael Perdue

**Affiliations:** Independent Researcher, Spring Green, WI 53588, USA; Independent Researcher, Indore 452005, M.P., India; Office of Indiana State Chemist, Purdue University, West Lafayette, IN 47907, USA; School of Earth and Atmospheric Sciences, Georgia Institute of Technology, Atlanta, GA 30332-0340, USA

## Abstract

**Background:**

Although humic substances are the principal ingredients in processed humic products, there has been no practical way to determine if a material is humified, allowing fake products to be used by farmers instead of genuine humic substances.

**Objective:**

To develop a test method using conventional laboratory techniques to determine if a material is humified.

**Method:**

A neutralized extract is prepared using the standardized extraction protocols specified in ISO 19822:2018(E). A portion of the extract is used to determine the concentration of dissolved organic matter on an ash-free basis. A portion of the remaining neutralized extract is diluted to a concentration of 30 mg/kg of dissolved organic matter and transferred to a quartz UV cuvette for ultraviolet-visible (UV-Vis) spectroscopy. UV-Vis absorbance is recorded over a wavelength range of 220–500 nm at 5 nm intervals. The absorbance data are normalized by conversion to scaled absorbance, which is compared to a reference scaled absorbance spectral curve for humic substances to determine if the tested material is humic or non-humic.

**Results:**

This method was able to differentiate legitimate humic substances from non-humic adulterants in a multiple-laboratory validation study (*P* ≤ 0.05).

**Conclusion:**

This method can differentiate humic from non-humic substances in materials intended to be used as ingredients in commercial humic products or for research.

**Highlights:**

This method uses common laboratory procedures and equipment.

Humic substances (HS) are complex heterogeneous organic materials that arise from biogeochemical reactions during the decay and transformation of plant and microbial organic matter into stable, extremely complex, dark-colored, heterogenous organic substances via a process called humification (1). This description reflects the difficulties of defining these materials, which is further confounded by the fact that there is no universally agreed-upon definition for the process of humification or the resultant humified (humic) materials.

Historically, humification has been defined as a continuous process that eventually reaches a stage dominated by heterogeneous amorphous substances, where none of the starting materials survive the transformation in their original chemical or physical form (2). This broad description has led to numerous interpretations of the humification process (3–7).

Because HS have no specific chemical structure (8), they are operationally defined as three principal fractions based on their aqueous solubility at various pH: humic acids,^a^ the fulvic fraction, and humin (9). All of the analytical methods that operationally define HS extracted from soils, natural water bodies, compost, humus, peat, and commercially significant geological deposits (10) assume the analytes of interest are derived from legitimate humified materials.

Currently, the ISO 19822:2018(E) standardized procedure for quantifying humic acids (HA) and the acidified hydrophobic fulvic acids (HFA), which is fractionated from the fulvic fraction, states that any material containing >0.75% (w/w) of elemental sulfur is not likely humic. Accordingly, any material failing that screen must be analyzed by Fourier transform infrared spectroscopy (FTIR), which is relatively expensive and requires an expert reviewer. As regulatory laboratories do not perform FTIR, regulators have no practical way to differentiate humic substances from non-humic materials.

The most common misrepresented humic material in the marketplace is fulvic acid. Use of the term “fulvic acid” (singular), which has no regulatory definition, is loosely defined by vendors as a humic substance that is soluble in both alkali and acid aqueous solutions. However, that operational definition includes many non-humic substances, such as mineral salts, polysaccharides, amino sugars, amino acids, mineral acids, low molecular weight organic acids, and certain carbohydrates (11), thus providing an opportunity for adulteration.

In the absence of a standardized test to determine if a material is humified, the geographical provenance of a material traceable to its origin is the only way to support a claim that a material is derived from humic substances. For example, all of the humic standard and reference materials provided by the International Humic Substances Society are named after the locale or the soil from which they are derived (1).

As alkaline extracts of humic substances contain relatively high concentrations of aromatic chemical structures and carboxylic functional groups (5), that characteristic has been extensively studied using ultraviolet-visible spectroscopy (UV-Vis) to characterize humified materials (12–17). The numerous functional groups associated with humic substances that respond to light as chromophores are primarily responsible for the higher degree of absorbance in the ultraviolet light region compared to the visible light region (13, 18).

Consequently, humic substances dissolved in alkaline aqueous solution have been characterized by UV-Vis spectra that exhibit decreasing light absorbance as the wavelength of light is increased, with a substantial decrease in absorbance in the visible light range of 400 to 700 nm (19, 20). The UV-Vis absorption spectra of humic substances from different sources are slightly different, but all humified materials generate the typical spectral curve of Figure 1 (14, 18).

**Figure 1.** UV-visible light absorbance spectral curve of humic material D2 extract, 30 mg/L concentration of dissolved organic matter in aqueous solution at pH 6.95 ± 0.05.

Numerous studies have explored the differences in UV-Vis light spectra of alkaline extracts of dissolved natural organic matter in an effort to establish UV-Vis indices of humification (15). The indices have been used to determine the degree of humification in soils (16), composts (21), the aquatic environment (22), and peat (5, 23), using either ratios of absorbance, molar absorption coeffcients, or absorbance relative to normalized carbon concentration at specific wavelengths of light (Table 1). As these indices demonstrate there are distinct differences between humified and non-humified materials, an investigation into their potential fit for purpose as standardized analytical methods was carried out. However, the authors were unable to correlate the results of the indices studies with the results of a preliminary study. It was decided the humification indices studies did not fit the purpose of the study because the indices studies:

**Table 1.** List of UV-Vis spectrographic indices for humified substances

Indices	Determination or calculation	Description	Reference
*E*_2_: *E*_3_	Ratio of absorbances at 250 and 365 nm (*A*_250_: *A*_365_)	Correlates with aromaticity and perhaps molecular weight.	Jiang et al., 2011 (16)
			Yakimenko et al., 2018 (17)
ε_280_	Molar absorption coefficient^a^ at 280 nm (L mol C _org_^−1^ cm ^−1^)	Correlates to concentration of aromatic substances related to molecular weight.	Chin, Aiken and O’Loughlin, 1994 (22)
ε_540_	Molar absorption coeffcient^a^ at 540 nm (L mol C _org_^−1^ cm ^−1^)	A peat humification index.	Zaccone et al., 2018 (23)
ε_465_	Molar absorption coeffcient^a^ at 465 nm (L mol C _org_^−1^ cm ^−1^)	Correlates with numerous humification indicators for soil humic acids.	Mahieu, Olk, and Randall, 2002 (24)
			Chen, Senesi, and Schnitzer, 1997 (25)
E_280/472_	UV-vis absorbance ratio of A_280 /A472_ nm	The proportion of lignins and other materials at the early stage of humification.	Yakimenko et al., 2018 (17)
E_280/665_	UV-vis absorbance ratio of A_280 /A665_ nm	Relationship of non-humified to humified material.	Yakimenko et al., 2018 (17)
SUVA_254_	Specific UV absorbance λ = 254 nm, A normalized relative to dissolved organic carbon (L mg C _org_^−1^ m ^−1^)	Correlated to aromaticity and compost maturity.	Weishaar et al., 2003 (26)
			Chen et al., 2017 (21)

a Some authors used the obsolete term molar extinction coeffect.

1. used various nonstandardized extraction procedures,
2. used absorbance data at wavelengths <280 and/or >350 nm to determine the degree of humification (16, 17, 27),
3. used dissolved elemental carbon as a reference,
4. typically used highly purified IHSS standards for comparison.

Preliminary studies were conducted by two laboratories to determine the optimum concentration of total dissolved organic matter (DOM) solution for reliable spectroscopy absorbance measurements. To avoid erratic readings at both the higher and lower wavelength ranges, numerous concentrations of DOM and ranges of final pH were tested. It was decided that the maximum light absorbance at 220 nm for DOM should not exceed 2.0, preferably about 1.5, to avoid inner filter effects and major shifts in pH due to overdilution (28).

The laboratories discovered that a concentration of 30 mg/L adjusted to 6.8–7.0 pH provided more consistent absorbance readings in the range of 250–700 nm, generating spectral curves that were consistent with other studies of DOM (19). The neutral pH range was chosen to optimize exposure of chromophores to light, avoiding collapse of DOM structures that occurs at low pH that would limit exposure of chromophores to light, or overexpanding structures at higher pH, exposing too many chromophores to light excitation (29). One standard method for measurement of UV absorbance of DOM stated that waters intended to be used in UV-Vis studies should not be <4 or >10 pH (30).

The first set of materials tested were mined humic ore materials, D2, D5, D6, D7, D8, D9, and two liquid humic acids extracts L1 and L2, derived from ore materials D8 and D2, respectively (Table 2). The absorbance spectral curves of all the humic materials were virtually identical to the spectral curve in Figure 1. Materials D9, L1, and L2 were later removed from the study because they were chemically processed by undisclosed proprietary methods. Non-humic materials D12, D13, and D14, which are materials that have been designated by US fertilizer regulators as adulterants in the marketplace, revealed visual differences in absorbance spectra between 300 and 400 nm.

**Table 2.** Materials used in the study

Material ID	Material	Source
D2	Humic ore	Southwestern United States
D5	Humic ore	Northcentral United States
D6	Humic ore	Western Canada
D7	Humic ore	Western United States
D8	Humic ore	Northcentral United States
D13	Soy protein	Grocery store
D14	Fulvic acid^a^	Internet purchase
M15	Molasses	Internet purchase
Compost^b^	Compost	United States Composting Council

a The product purchased was clearly labeled “fulvic acid,” but upon further analysis, it was actually a lignosulfonate.

b The compost material was supplied to laboratories identified as “compost”; therefore, there is no ID number.

The absorbance data generated by the laboratories in the study were highly variable, which is typical for extracted humic substances (18) due to variation within the heterogeneous materials and operator error. To normalize the absorbance data, scaled absorbance was incorporated. The wavelength of 290 nm was chosen because it has been used in a previous study (31) to avoid potentially erroneous absorbance data generated in the range of 250–300 nm from the presence of inorganic ions, such as nitrates, nitrites, bromides (22, 30), lignins (13), and numerous aromatic, alkene, and alkyne non-humic substances that absorb UV in that range (20).

## Experimental

The object of this study was to test the proposition that ultraviolet spectroscopy of alkaline extracts of organic matter can be used to determine if a material is humic or non-humic using standardized extraction procedures and common laboratory equipment. A multiple-laboratory collaborative study was implemented to measure the UV-Vis absorbance of both humic and non-humic substances in alkali extracts. Five humic ores supplied by members of the Humic Products Trade Association from five different geological deposits were analyzed using the alkaline extraction procedures in the international standard ISO 19822:2018 (E). The study was performed by 14 analysts from nine different laboratories, replicating the analyses three times for each humic and non-humic material.

### Reagents

All chemicals are ACS certified.

- *NaOH pellets.—*Formula weight 39.997 g/mol, purity ≥97%, CAS 1310-73-2.
- *Concentrated HCl.—*Formula weight 36.46 g/mol, 34 to 37% concentration, CAS 7647-01-0.
- *Nitrogen gas.—*≥99.99% purity.
- *Deionized water or Milli-Q water.*

### Quality Control Material

The quality control material (QCM 1.0) used in this study was prepared by following the experimental procedure using material D2 as the raw material to produce a neutralized extract, which was diluted to 30 mg/kg. The concentration of DOM in the QCM 1.0 was confirmed by an independent laboratory who did not participate in the study.

### Equipment

- *Analytical balance.*—With 220 g capacity and readability to 0.0001 g (Mettler Toledo XSR204 or equivalent) and top-loader balance with readability to 0.01 g.
- *General purpose heating and drying oven.*—Precision ± 3°C, (Isotemp™, Fisherbrand™, or equivalent).
- *Centrifuge.*—Minimum relative centrifugal force 1500 × *g* (Beckman Coulter, J6-MI or equivalent).
- *Magnetic stir plates (VWR 365 or equivalent) and stir bars.*
- *pH meter with probe.—*pH range 0–14, resolution pH 0.01.
- *Spectrophotometer.—*Dual-beam or double-beam 200 to 900 nm, 1.0 nm spectral bandwidth with wavelength accuracy of ≤ ± 1 nm and repeatability of ≤0.5 nm (Evolution 60S, Thermo Scientific or equivalent).
- *Quartz cuvettes.—*Standard rectangular with 10 mm pathlength (Z276669, Sigma-Aldrich, or equivalent).
- *Muffle furnace.—*(Lindberg/Blue M^TM^ BF51732C-1 or equivalent).
- *Adjustable (electronic or manual) volumetric pipets*.—Capable of volumes 100–1000 µL.

### Glassware

- *Erlenmeyer flasks.—*500 mL.
- *Graduated cylinder.—*500 mL.
- *Beakers.—*500 mL.
- *50 mL wide-form porcelain crucibles.*

### Other Miscellaneous Laboratory Items

- Weighing boats or weighing papers, Parafilm™, 250 mL centrifuge bottles; desiccator; disposable transfer pipets for pH adjustment; and 250 mL storage bottles.

## Experimental Procedure

### Preparation of Crucibles

*(1)* Prepare two 50 mL crucibles for dissolved organic matter determination. If using new crucibles, wash them with acetone and then dry them in an oven at 105°C for 2 h. If the crucibles have been used previously, wash in acetone, and then place them in a furnace at 575°C for 2 h. Cool the crucibles in a desiccator to room temperature. Leave the crucibles in the desiccator until Step 7.
*Note:* For Step 7, wide-form crucibles provide quicker drying time than high-form crucibles.
*(2)* Preparing the analytical sample:
*(a)* For solid laboratory samples: crush the entire laboratory sample into a fine uniform powder using a mortar and pestle. Pass the sample through a 74 μm (200 mesh) screen.
*(b)* For liquid laboratory samples: thoroughly mix the laboratory sample by shaking the container as received for approximately 1 min. Do not pour an aliquot of the liquid from the container. Instead, insert an open tube (thief) or straw as deep as possible into the container to remove the liquid.^b^ Proceed to Step 3 immediately to reduce settling of suspended material.
*(3)* Alkaline extract: weigh out 1.00 ± 0.05 g test portion increment of the analytical sample prepared in Step 2 in a 500 mL Erlenmeyer flask containing a magnetic stir bar. Add 200 mL of 0.05M NaOH solution. Evacuate the head space with N_2_, cover the flask with Parafilm™ (or equivalent), and then stir constantly at 300–400 rpm for 1 h.
*Note:* Prepare a sufficient amount of 0.05 molarity NaOH (e.g., 2 L) for Step 3 and Step 12. To make 2 L of 0.05 molarity NaOH, add approximately 1000 mL of DI or Milli-Q water into a 2 L volumetric flask, add 4 g of NaOH pellets, and bring to final volume with DI or Milli-Q water.
*Note:* Stir all of the extractions as uniformly as possible. Use the same size stir bar in Step 3 for all extractions. If multiple extractions are being performed using multiple stir plates simultaneously, be sure to use the same size stir bar.
*(4)* Transfer the alkaline extract solution from Step 3 to a 250 mL centrifuge bottle, and then centrifuge at 3900 × *g* for 15 min.
*(5)* Neutralized extract solution: Carefully decant the centrifuged alkaline extract solutions into a 500 mL beaker containing a clean stirring bar, and then adjust the solution dropwise with a disposable transfer pipet first to a pH between 7.5 and 8 using 6 molarity HCl and to a final pH of 6.8–7.0 using 0.6 molarity HCl while stirring in a fumehood.
*Note:* To make 500 mL of 6 molarity HCl, add 246 mL concentrated HCl to 125 mL DI or Milli-Q water in a 500 mL volumetric flask; bring to final volume with DI or Milli-Q water. To make 500 mL of 0.6 molarity HCl, add 50 mL of 6 molarity HCl to 125 mL DI or Milli-Q water in a 500 mL volumetric flask, and bring to final volume with DI or Milli-Q water.
*Caution:* Perform Steps 6 and 7 immediately.
*(6)* Transfer the neutralized extract to a 250 mL centrifuge bottle and centrifuge at 3900 × *g* for 15 min to separate insoluble material. After centrifugation is complete, decant the solution into another 250 mL centrifuge bottle, or a 250 mL bottle with a lid if storing overnight.
*(7)* Using the prepared crucibles from Step 1, remove one crucible from the desiccator, weigh and record the weight of the crucible as crucible weight (g) to four decimal places, and then immediately transfer a 15 ± 0.10 g aliquot of the centrifuged neutralized extract to the crucible. Record the initial weight of the crucible + neutralized extract solution to four decimal places as the initial sample + crucible weight (g). Place the crucible in a drying oven at 62 ± 3°C until a constant mass is obtained. Repeat Step 7 with a second crucible.
*Caution:* Do not allow the oven temperature to exceed 65°C. Exceeding 65°C will decompose natural organic matter.
*Note:* As the drying time may exceed 8 h, it is advisable to dry the solution overnight.

### Quantification of Organic Matter in the Neutralized Extract Solution

*(8)* Remove the crucibles from the drying oven and place them in a desiccator after a constant mass is obtained. Cool the crucibles to room temperature. This usually takes 30 to 60 min. Weigh and record weight each Crucible + Dried Matter as *Crucible + Dried Matter Weight (g) to* four decimal places.
*(9)* Determine ash content of the dried matter by combusting Crucibles + Dried Matter in a preheated furnace for 2 h at 575°C. If any solid clumps form during ashing, carefully break up the clumps using a glass rod. Do not use a metal rod. After achieving constant weight, remove the crucibles and ash from the furnace and place them in a desiccator to cool to room temperature. When cooled, weigh each crucible and record as *Crucible + Ash Weight (g)* to four decimal places.
*(10)* Calculate the ash-free organic matter content in the neutralized extract solution using the formula below. Record the average of the two results. Discard the ash when finished with this step.
  $$\begin{array}{c} \text{Ash}-\text{Free Organic Matter in Neutralized Extract Solution}\;\\ \left(\text{mg}/\text{kg}\right)=1,000,000\;\times \;[\left(\text{Crucible}+\text{Dried Matter Weight}\right)\;\\ –\;\left(\text{Crucible}+\text{Ash Weight}\right)]/\\ \left[\left(\text{Initial Sample}+\text{Crucible Weight}\right)-\left(\text{Crucible Weight}\right)\right] \end{array}$$

### Preparing the UV-Vis Test Solution

*(11)* Using the organic matter concentration calculated in Step 10, determine the mass of the neutralized extraction needed from Step 6 for dilution to achieve a final concentration of 30 mg/kg of dissolved organic matter in a UV-Vis test solution for UV-Vis scanning.

### Example Calculation

If a neutralized extract has an ash-free organic matter concentration of 5000 mg/kg as determined in Step 10 above, and if the amount of UV-Vis test solution needed to sufficiently fill the quartz cuvette for scanning is 20 g, then the mass (M) of neutralized extract to achieve a concentration of 30 mg/kg organic matter in the test solution is: 


$$\begin{array}{c} \left(5,000\;\text{mg}/\text{kg}\right)\;\times \;M=\left(30\;\text{mg}/\text{kg}\right)\;\times \;\left(20\;g\right)\\ M=0.12\;g \end{array}$$

In this case, 0.12 g of neutralized extract solution would be weighed with an analytical balance and diluted to a final mass of 20.0 ± 0.1 g using deionized or Milli-Q water to prepare the test sample for UV-Vis analysis.

*Note:* Use an adjustable pipet (for example, 100–1000 µL) for the neutralized extract solution to get better accuracy for the creation of the UV-Vis test solution and weigh the mass using an analytical balance. For example, pipet 115–125 µL extract solution to obtain 0.12 ± 0.005 g neutralized extract solution.

### Scan

*Caution:* Use standard quartz UV cuvettes with 1 cm pathlength. Do not use plastic or glass cuvettes.

*Note:* Clean the quartz cuvettes before and after use with fresh deionized or Milli-Q water.

*(12)* Baseline scan: Prepare a blank neutralized extract. Using the 0.05M NaOH solution prepared in Step 3, adjust the solution dropwise with a disposable transfer pipet to a pH between 7.5 and 8 using 6M HCl, and then to a final pH of 6.9 ± 0.1 using 0.6M HCl while stirring in a fumehood. Follow the operating procedure for your instrument to establish baseline scan data 220–500 nm for the blank extract.
*Note:* Although the scan is from 220 to 500 nm, only 290–330 nm is used for comparison to the humic standard curve.
*(13)* Quality control material calibration: Shake the bottle of quality control material (QCM 1.0) for 30 seconds prior to transferring an aliquot to a cuvette. The QCM 1.0 does not require any sample preparation; use as received. Rinse a clean cuvette with a small aliquot of QCM 1.0. Fill the cuvette with the QCM 1.0*.* Measure the UV-Vis light absorbance over a wavelength range of 220–500 nm at 5 nm intervals accurate to four decimal places (0.0000 nm).
*(14)* *Note:* Steps 14 and 16 require the Humic Dashboard spreadsheet in the Supplemental Information.
  Copy and paste the absorbance results for material QCM 1.0 in the range of 290–330 nm only into the Humic Dashboard tab labeled “Sample Testing.” If the result reads “Sample is Humic,” proceed to Step 15. If the result is “Sample is Non-Humic,” review all of the steps to find the error.
*(15)* UV test solution scan: Clean the quartz cuvettes with fresh deionized or Milli-Q water. Rinse the cuvette with a small aliquot of the test solution. Transfer a test portion of the UV-test solution prepared in Step 11 to the cuvette for UV-Vis absorbance measurements. Measure absorbance over a wavelength range of 220–500 nm at 5 nm intervals.
*Note:* For quartz cuvettes, handle the top portion of the non-optical side only. Rinse with deionized or Milli-Q water completely, and store in the appropriate case when not in use.
*(16)* Copy and paste the absorbance data for the range of 290–330 nm into the Humic Dashboard tab labeled Sample Testing. If the Dashboard returns “Sample is Non-Humic,” repeat the entire procedure to confirm the first result.

## Results

### Scaled Absorbance

Scaled absorbance normalizes the UV-Vis spectra internally, irrespective of dilution, and reduces interference from the presence of non-chromophoric organic matter, thus allowing the distribution of chromophores in different solutions of dissolved organic matter to be compared (31).

To calculate scaled absorbance, the absorbance data were zeroed by subtracting the minimum absorbance value from all values in the absorbance set of data to obtain zeroed absorbance, thus eliminating dilution effects on absorbances obtained at the lower limits of detection. Scaled absorbance was calculated by dividing all the zeroed absorbance values by the zeroed absorbance at wavelength of 290 nm.

Initially, scaled absorbance in the range of 220–700 nm for humic substances was used; however, scaled absorbance values of humic-containing materials were normally distributed only in the range of 295–325 nm (Table 3 and Supplemental Table 1). None of the scaled absorbance data >350 nm were normally distributed. Consequently, the humic standard curve was produced by averaging the scaled absorbance data for all the humic samples corresponding to the 290–330 nm wavelengths (Figure 2).

**Figure 2.** The humic standard curve 290–330 nm for humic substances, which is the mean of the scaled absorbance for the total population from 290 to 330 nm measured at 5 nm intervals.

**Table 3.** Results of ShapiroWilk test performed on the scaled absorbance data for all humic samples

Wavelength, nm	295	300	305	310	315	320	325
N	194	194	194	194	194	194	194
Mean	0.8682	0.7387	0.6115	0.4845	0.3600	0.2375	0.1172
Std Dev	0.0028	0.0031	0.0033	0.0031	0.0026	0.0026	0.0025
CV	0.32%	0.42%	0.55%	0.66%	0.73%	1.09%	2.09%
p	0.1998	0.2913	0.3996	0.4764	0.6087	0.1773	0.000012
W	0.99	0.99	0.99	0.99	0.99	0.99	0.96

### Scaled Absorbance Difference

A scaled absorbance difference graph was generated by plotting the difference between the standard curve and the scaled absorbance data for non-humic substances by subtracting the scaled absorbance of test solutions from the scaled absorbance in the standard curve. Visually, the plots for the scaled absorbance difference suggest that there is a measurable difference between test solutions of non-humified materials and the humic standard curve in the ultraviolet wavelength range (Figure 3).

**Figure 3.** Scaled absorbance difference relative to the humic standard curve for humified materials (orange line at 0.0) and non-humified materials at 30 mg/L concentration of dissolved organic matter (DOM), suggesting there is a measurable difference between humic and non-humic materials.

### Statistical Procedures

A statistical methodology was developed intended to differentiate between the humic and non-humic materials using UV-Vis spectral absorbance data of the humic neutralized extracts. This identification is based on scaled absorbance (normalized absorbance data), scaled absorbance difference, and the square of sum of the scaled absorbance difference (SSSAD) between humic and non-humic extracts. Scaled absorbance and SSSAD values were derived from the absorbance data in the following steps:

- Zeroing the absorbance data
- Evaluation of scaled absorbance data
- Finding the scaled absorbance difference
- Finding the sum of scaled absorbance difference values at different wavelengths
- Finding the squared values of sum of scaled absorbance difference (SSSAD) calculated in previous step

The above steps were performed using the humic standard curve as reference (Figure 2). To get an estimate of standard deviation in the humic standard curve data, the standard error of the mean (SEM) of the humic standard curve was calculated. A variation of 2×SEM was applied to the mean of scaled absorbance data indicating variations <0.2%. Therefore, the mean of scaled absorbance data was used as a standardized data set to evaluate the scaled absorbance difference. Scaled absorbance difference between the values in the standard curve and the values for non-humic containing test solutions was used to calculate the SSSAD, a unitless quantity achieved by squaring the sum of scaled absorbance difference values at each wavelength.

The maximum values of SSSAD for humic solutions were found to be 0.001055152, while minimum values of SSSAD for non-humic solutions were 0.022867392. The mean value of those differences (0.01) was defined as the boundary between humic and non-humic substances. Any value above 0.01 was hypothesized to indicate the material tested is non-humic (Figure 4).

**Figure 4.** Summary of hypothesis testing of humic and non-humic samples using square of sum of the scaled absorbance difference (SSSAD) demonstrating all non-humic samples tested penetrated the boundary of 0.01 SSSAD.

To test the hypothesis, one-sample Student’s *t*-test was applied to test the significant difference between the SSSAD values of humic and non-humic materials (*P* ≤ 0.05). For each humic and non-humic material, the mean was calculated for all the materials tested by different laboratories. For the comparison population mean was fixed as 0.01. The hypothesis testing was based on the *P*-value. The hypotheses tested were H0: ≤0.01 (The material tested is humic), H1: >0.01 (the material tested is non-humic). Table 4 is an example of the hypothesis testing result; D2 tested humic, and material D14 tested non-humic. Material D14 is a lignosulfonate, which is a common adulterant.

**Table 4.** Example of a one-sample *t*-test analysis for (a) humic material D2, (b) non-humic material D14 (the number after the letter “L” is the laboratory ID)

(a)										
Humic data (sample D2)								Analysis		Testing
	Rep1	Squared	Rep2	Squared	Rep3	Squared	Sq avg	Sample mean	0.0002	Hypothesis testing
D2L3	−0.002848	0.000008	−0.032483	0.001055	−0.025422	0.000646	0.000570	Pop mean	0.01	H0: ≤0.01 (The material tested is humic)
D2L3a	−0.018554	0.000344	−0.026548	0.000705	−0.029306	0.000859	0.000636	Std dev	0.000236961	
D2L4	−0.019744	0.000390	−0.025905	0.000671	−0.015125	0.000229	0.000430	Count	12	H1: >0.01 (The material tested is non-humic)
D2L5	0.004066	0.000017	0.002655	0.000007	0.002915	0.000008	0.000011	dof	11	
D2L5a	0.003120	0.000010	−0.005485	0.000030	0.001353	0.000002	0.000014	num	−0.0098	Fail to reject
D2L6	−0.009592	0.000092	−0.006579	0.000043	−0.016567	0.000274	0.000137	denom	6.84047E-05	
D2L8	−0.003106	0.000010	0.001726	0.000003	0.000822	0.000001	0.000004	t-stat	−143.444666	
D2L9	0.004249	0.000018	0.010004	0.000100	0.012950	0.000168	0.000095	t-critical	−1.795884819	
D2L10	−0.005674	0.000032	0.001912	0.000004	−0.005023	0.000025	0.000020	p	1	Sample is humic
D2L10a	0.001737	0.000003	−0.004547	0.000021	0.003280	0.000011	0.000011			
D2L11	0.003042	0.000009	−0.001458	0.000002	−0.004787	0.000023	0.000011			
D2L11a	−0.018156	0.000330	−0.018727	0.000351	−0.016044	0.000257	0.000313			

(b)										
Non-Humic data (material D14)								Analysis		Testing
	Rep1	Squared	Rep2	Squared	Rep3	Squared	Sq avg	Sample mean	1.099504926	Hypothesis testing
D14L1	−1.125982249	1.267836025	−1.069876154	1.144634985	−1.089394273	1.186779882	1.199750297	Pop mean	0.01	H0: ≤0.01 (The material tested is humic)
D14L5	−1.061833199	1.127489743	−0.995210947	0.99044483	−1.052627215	1.108024054	1.075319542	Std dev	0.131011475	
D14L7	−1.064150903	1.132417144	−1.073406436	1.152201377	−1.134573438	1.287256886	1.190625136	Count	6	H1: >0.01 (The material tested is Non humic)
D14L8	−0.990731664	0.98154923	−0.95974184	0.921104399	−0.916263579	0.839538946	0.914064192	dof	5	
D14L9	−1.122145932	1.259211492	−1.112892792	1.238530367	−1.099807883	1.209577379	1.235773079	num	1.089504926	The null hypothesis is rejected
D14L10	−0.982123	0.964565588	−0.986371886	0.972929498	−1.003492327	1.006996851	0.981497312	denom	0.053485211	
								t-stat	20.37020917	
								t-critical	−2.015048373	
								P	2.63723E-06	Sample is Non-Humic

## Discussion

To develop a standardized quantitative analysis, all steps in the procedure must be standardized to increase the likelihood of repeatability. As the alkaline extraction protocols in ISO 19822 have been validated, those protocols fit the purpose of this experiment.

Regarding the four points made about using humic indices in the introductory section above, points 2 and 3 refer to the debate of the degree to which UV absorbance spectroscopy of dissolved organic matter at <280 nm is influenced by non-humic substances (26), and whether all humified substances absorb in visible light, especially >465 nm (19). Additionally, as almost all regulatory laboratories lack the equipment needed to determine dissolved elemental organic carbon, dissolved organic matter was chosen as the analyte.

Furthermore, the indices studies used either IHSS humic acids or IHSS fulvic acids standard and reference materials developed by the International Humic Substances Society (IHSS). However, they are idealized, homogenized models derived from various sources to meet specific classifications for comparative purposes. They do not represent the complexity of natural organic matter found in real-life commercial humic ingredients, and there are 33 different IHSS standard and reference materials, with various ash and chemical composition (32).

To meet the purpose of this study, a quality control material (QCM1.0) reference material was prepared by means of the protocols in the experimental procedure. The mean SSSAD for the QCM 1.0 was 0.00002, well within the SSSAD limits of 0.01 for all humic substances tested (*n* = 53, residuals <4.2%).

Statistically, the data for scaled absorbance values of humic containing solutions were normally distributed only in the range of 295–325 nm (Table 3). All data >350 nm were not normally distributed. The results are consistent with the relative concentration of chemical moieties responsible for absorbance by humic substances in the ultraviolet range from 200 to 400 nm, which are well defined, dominated by conjugated aliphatic, aromatic, and carboxylic electron systems (19, 20). The pronounced differences between humic and non-humic substances in absorption between 330 and 400 nm are due to electron transfer bands of phenolic and hydroxyl functional groups associated with substituted benzene ring chromophores that are more abundant in humic substances (13, 22) relative to non-humic substances.

Eliminating absorbance values at wavelengths >400 nm is further justified because it is difficult to determine the identity of chromophores at higher wavelengths (19). The differences in absorbance at higher wavelengths are very sensitive to pH due to changes in structural conformation of humic substances (22), generating a higher degree of variation in the context of analytical results. Furthermore, non-humic substances, such as carotenoids, amino acids, proteins, and saccharides, absorb light in the 400–700 nm range (19), which do not necessarily follow the Beer-Lambert law due to interactions among macromolecular chromophores (33).

For regulatory purposes, extracts of naturally occurring humic substances from mined sources are more likely to represent the analytes of interest rather than highly purified reference materials because mined materials are nonsynthetic, naturally occurring, unprocessed materials that contain both humic acids and hydrophobic fulvic acids as defined by ISO 19822, as well as unknown substances that have gone through the humification process.

Supportive evidence for this theory emerged from this study and two prior studies. In this study, two liquid and one solid humic acids materials were reviewed as potential reference materials because they contain both humic acids and hydrophobic fulvic acids. However, they were not used as reference materials because they were derived from mined ores through unspecified proprietary processes that may have changed their chemistry. Nonetheless, they passed this test method as “humic.” Furthermore, most of the materials used in this study were the same as those materials used to develop the ISO 19822 standard method and the Lamar et al. (34) quantitative analytical procedures, where the study materials represented a range of sources and concentrations for both humic acids and hydrophobic fulvic acids. Both studies reported significant concentrations of both humic acids and hydrophobic fulvic acids in all the mined ores.

This method does not include humin, which is operationally defined as the insoluble portions of humic substances; humin is removed in Step 6 of the experimental procedure. However, this method does capture the operationally defined humic acids and hydrophobic fulvic acids (35), and numerous unknown substances that have gone through the humification process, which is consistent with the composition of commercial humic products. Therefore, ultraviolet absorbance measurement of alkaline extracts of humic substances is an aggregate measure of all dissolved organic matter in an analytical sample. Additionally, there were no reports of any substances (humic acids precipitating out of the neutralized extract).

However, it should be pointed out that this method eliminates interferences from non-humic substances that are also present in typical commercial products, especially iron (26), harmonized with the ash-free basis protocols in ISO 19822.

This procedure does not specifically identify humic acids or hydrophobic fulvic acids; instead, it determines if a laboratory sample is humified, which is an all-encompassing characteristic of humified materials, not restricted to the operationally defined substances humic acids and hydrophobic fulvic acids. It is essentially a “sniff test” that regulators can perform in their own laboratories, while providing an opportunity to defend their results by enlisting referee laboratories in the analytical community if necessary.

The most common example of mislabeling of humic substances in the marketplace is fulvic acid.^c^ As these products are operationally defined by vendors as purported humic substances that are soluble in both alkaline and acid aqueous media, these products have a wider appeal than humic acids because they have a wider range of aqueous solubility, making them more versatile and therefore commanding a higher price point.

Each laboratory in the study had the option to pick a material that in their opinion is being used in commerce as a fake humic substance. Eight non-humic optional (NHO) materials were tested: two seaweed extracts, three commercial products labeled fulvic acid, and three molasses products. The test method determined all the NHO materials were non-humic (Table 5).

**Table 5.** The results of hypothesis testing on non-humic optional (NHO) materials chosen by laboratories 1, 5, 7, 8, 9, and 10 as suspected to be false humic materials

	Non-humic optional materials							
		Rep1	Squared	Rep2	Squared	Rep3	Squared	Sq avg
Seaweed Extract	NHOL1	−0.416263579	0.173275367	−0.219323936	0.048102989	−0.216440492	0.046846486	0.089408281
Molasses 1	NHOL5	−0.325354488	0.105855543	−0.616263579	0.379780799	−0.416263579	0.173275367	0.219637236
Seaweed extract 2	NHOL7	−0.613233276	0.376055051	−0.680969461	0.463719407	−0.61029343	0.37245807	0.404077509
Commercial fulvic acid 2	NHOL8	−1.511740966	2.285360748	−1.530007655	2.340923423	−1.548494984	2.397836715	2.341373629
Fake fulvic acid product 1	NHO9	−1.725655844	2.977888092	0.292069755	0.085304741	0.295798678	0.087496858	1.050229897
Molasses 2	NHO10	−1.193499417	1.424440859	−1.03519527	1.071629246	−1.111621284	1.235701878	1.243923994

Analysis		Testing
Sample mean	0.891441758	Hypothesis testing
Pop mean	0.01	H0: ≤0.01 (The material tested is humic)
Std dev	0.846624209	
Count	6	H1: >0.01 (The material tested is non-humic)
dof	5	
num	0.881441758	The null hypothesis is rejected
denom	0.345632886	
t-stat	2.55022538	
t-critical	−2.015048373	
p	0.025626001	Sample is non-humic

Only two laboratories tested the compost material. The test results indicate that the compost material was non-humic. With only two results, it is not possible to determine why the compost tested non-humic.

Future studies should include the ability to detect humic and non-humic substances added to liquid fertilizers and the determination of detection limits.

## Conclusions

By harmonizing the alkaline extraction protocols with ISO 19822, this method reproduces the standardized operational definition of humic substances. Adjusting the alkaline extract to pH 6.9, instead of pH 1, the extraction method recovers humic acids and fulvic fractions, as well as unknown humified materials. Ultraviolet spectroscopy of the alkaline extracts identified a wide range of non-humic (fake) from legitimate humic materials by establishing a standard scaled absorbance spectral curve for humic substances.[Fn qsad001-en4]

## Supplementary Material

qsad001_Supplementary_Data

## Footnotes

a The plural “humic acids” is appropriate because humic acids are a continuum of extremely complex chemical moieties making up humic substances, with no specific structure or molecular weight. There is no particular point where a single molecule of humic acid (singular) exists.

b AAFCO, 2018. GOOD Test Portions: Guidance on Obtaining Defensible Test Portions. Laboratory Sampling Working Group, Association of American Feed Control Officials, Champaign, IL, https://www.aafco.org/Portals/0/SiteContent/Publications/GoodTP_final_web.pdf?v3. Accessed August 4, 2022.

c The singular usage of the term “fulvic acid” typically appears on labels that have not gone through regulatory review because “fulvic acid” is not an official AAPFCO term.

d Compendium of Chemical Terminology, Gold Book. International Union of Pure and Applied Chemistry, Version 2.3.3, 2014-02-24.

## References

[1] IHSS (2019) What are humic substances? http://humic-substances.org/what-are-humic-substances-2 (accessed September 3, 2022)

[2] Hayes M.H.B. , SwiftR.S. (2018) J. Soils Sediments18, 1212–1231. doi:10.1007/s11368-016-1636-6

[3] Kononova M.M. (1966) Soil Organic Matter: Its Nature, Its Role in Soil Formation and in Soil Fertility, 2nd Ed. Pergamon Press, Oxford, UK

[4] Hayes M.H.B. , SwiftR.S. (1978) in The Chemistry of Soil, GreenlandD.J., HayesM.H.B. (Eds), Wiley, Chichester, UK, pp 179–320

[5] Stevenson F.J. (1994) Humus Chemistry: Genesis, Composition, Reactions, 2nd Ed. John Wiley & Sons, New York, NY.

[6] Piccolo A. (2001) Soil Science166, 810–832

[7] US Geological Survey Scientific Investigations Report 2004–5121 (2004) Evaluation of conceptual models of natural organic matter (humus) from a consideration of the chemical and biochemical processes of humiﬁcation, https://pubs.usgs.gov/sir/2004/5121/pdf/sir2004-5121.pdf (accessed September 28, 2022)

[8] Ghabbour E.A. , DaviesG. (2001) Humic Substances: Structures, Models and Functions, Royal Society of Chemistry, Cambridge, UK.

[9] Stevenson F.J. (1965) in Methods of Soil Analysis, Part 2, Chemical and Microbiological Properties, BlackC.A. (Ed), American Society of Agronomy, Madison, WI, pp 1414–1417

[10] Liem E.L. (2021) Low-Rank Coal Applications in Agriculture: Humic Analysis, Products, and Performance, John Wiley & Sons, Hoboken, NJ

[11] Schnitzer M. (1982) in Methods of Analysis, Part 2, Chemical and Microbiological P*roperties*, 2nd Ed. American Society of Agronomy, Inc., PageA.L. (Ed), Soil Science Society of America, Inc., Madison, WI, pp 581–594

[12] Jarukas L. , IvanauskasL., KasparavicieneG., BaranauskaiteJ., MarksaM., BernatonieneJ. (2021) Molecules26, 2995. doi: 10.3390/molecules2610299534069989 PMC8157823

[13] Martin-Neto L. , MiloriK., Da SilvaW., SimoesM. (2009) in Biophysico-Chemical Processes Involving Natural Nonliving Organic Matter in Environmental Systems, SenesiN., XingB., HuangP.M. (Eds), John Wiley & Sons, Hoboken, NJ, pp 651–727

[14] Korshin G.V. , LIC., BenjaminM. (1997) Water Res. 31, 1787–1795

[15] Fuentes M. , González-GaitanoG., García-MinaJ. (2006) Org. Geochem. 37, 1949–1959. doi: 10.1016/j.orggeochem.2006.07.024

[16] Jiang J. , YuH., XiB., MengF., ZhouY., LiuH. (2011) Soil Res.49, 670–679. doi:10.1071/SR11213

[17] Yakimenko O. , KhundzhuaD., IzosimovA., YuzhakovV., PatsaevaS. (2018) J. Soils Sediments18, 1279–1291. doi: 10.1007/s11368-016-1528-9

[18] Kumada K. (1987) Chemistry of Soil Organic Matter, Japan Scientific Societies Press, Elsevier, Tokyo, Japan

[19] Bloom P.R. , LeenheerJ.A. (1989) in Search of Structure, HayesM.H.B., MacCarthyP., MalcolmR.L., SwiftR.S. (Eds), John Wiley & Sons, Hoboken, NJ, pp 409–446

[20] Baes A.U. , BloomP.R. (1990) Soil Sci. Soc. Am. J. 54, 1248–1254

[21] Chen Y. , JiangZ., ZhangX., CaoB., YangF., WangZ., ZhangY. (2017) J. Environ. Qual.46, 1489–1499. doi:10.2134/jeq2017.07.026029293826

[22] Chin Y.P. , AikenG., O'LoughlinE. (1994) Environ. Sci. Technol.28, 1853–1858. doi:10.1021/es00060a01522175925

[23] Zaccone C. , PlazaC., CiavattaC., MianoT., ShotykW. (2018) Earth-Sci. Rev. 185, 163–178. doi:10.1016/j.earscirev.2018.05.017

[24] Mahieu N. , OlkD.C., RandallE.W. (2002) J. Environ. Qual.31, 421–43011931429

[25] Chen Y.N. , SenesiN., SchnitzerM. (1977) Soil Sci. Soc. Am. J. 41, 352–358

[26] Weishaar J.L. , AikenG.R., BergamaschiB.A., FramM.S., FujiiR., MopperK. (2003) Environ. Sci. Technol.37, 4702–4708. doi:10.1021/es030360x14594381

[27] Peuravuori T. , PihlajaK. (1997) Anal. Chim. Acta337, 133–149

[28] Kothawala D.N. , MurphyK., StedmonC., WeyhenmeyerG., TranvikL. (2013) Limnol. Oceanogr. Methods11, 616–630. doi:10.4319/lom.2013.11.616

[29] Pace M.L. , RecheI., ColeJ., Fernandez-BarberoA., MazuecosI., PrairieY. (2012) Biogeochemistry108, 109–118. doi:10.1007/s10533-011-9576-0

[30] Eaton A. (1995) J. Am. Water Works Assoc. 87, 86–90. doi:10.1002/j.1551-8833.1995.tb06320.x

[31] Bianchi T.S. , CookR.L., PerdueE.M., KolicP.E., GreenN., ZhangY., SmithR.W., KolkerA.S., AmeenA., KingG., OjwangL.M., SchneiderC.L., NormandA.E., HetlandR. (2011) Mar. Environ. Res.72, 248–257. doi:10.1016/j.marenvres.2011.09.00722000271

[32] Elemental Composition and Stable Isotopic Ratios of IHSS Samples, https://humic-substances.org/elemental-compositions-and-stable-isotopic-ratios-of-ihss-samples/ (accessed October 1, 2022)

[33] Piccolo A. , ConteP., CozzolinoA. (2000) in Humic Substances: Versatile Components of Plants, Soil and Water, GhabbourE.A., DaviesG. (Eds), Royal Society of Chemistry, Cambridge, UK, pp 111–124

[34] Lamar R. , OlkD., MayhewL., BloomP.R. (2014) J. AOAC Int.97, 721–730. doi:10.5740/jaoacint.13-39325051616

[35] AAPFCO (2022) in Official Publication, 75th Ed. McMurryS. (Ed), Association of American Plant Food Control Officials, West Lafayette, IN, pp 86–118

